# The Role of SliTrk5 in Central Nervous System

**DOI:** 10.1155/2022/4678026

**Published:** 2022-07-14

**Authors:** Yan Liu, Linming Zhang, Rong Mei, Mingda Ai, Ruijing Pang, Di Xia, Ling Chen, Lianmei Zhong

**Affiliations:** ^1^Department of Neurology, The First Affiliated Hospital of Kunming Medical University, Kunming, Yunnan 650032, China; ^2^Yunnan Provincial Clinical Research Center for Neurological Disease, Kunming, Yunnan 650032, China; ^3^Department of Neurology, The First People's Hospital of Yunnan Province, Kunming, Yunnan 650034, China

## Abstract

SLIT and NTRK-like protein-5 (SliTrk5) is one of the six members of SliTrk protein family, which is widely expressed in the central nervous system (CNS), regulating and participating in many essential steps of central nervous system development, including axon and dendritic growth, neuron differentiation, and synaptogenesis. SliTrk5, as a neuron transmembrane protein, contains two important conservative domains consisting of leucine repeats (LRRs) located at the amino terminal in the extracellular region and tyrosine residues (Tyr) located at the carboxyl terminal in the intracellular domains. These special structures make SliTrk5 play an important role in the pathological process of the CNS. A large number of studies have shown that SliTrk5 may be involved in the pathogenesis of CNS diseases, such as obsessive-compulsive-disorder (OCD), attention deficit/hyperactivity disorder (ADHD), glioma, autism spectrum disorders (ASDs), and Parkinson's disease (PD). Targeting SliTrk5 is expected to become a new target for the treatment of CNS diseases, promoting the functional recovery of CNS. The purpose of this article is to review the current research progression of the role of SliTrk5 in CNS and its potential mechanisms in CNS diseases.

## 1. Introduction

Increasing evidence has identified that SliTrk5 can modulate many important stages of central nervous system development, including axon and dendritic growth, neuron differentiation, and synaptogenesis, which may affect the pathological mechanism of many central nervous system diseases [1]. The expression of SliTrk5 is highly restricted to neural tissue of CNS, compared with various systems throughout the body. It has two conserved domains: leucine repeats (LRRs) located at the amino terminal in the extracellular region and tyrosine residues located at the carboxyl terminal in the intracellular domains. The LRR domain is highly similar to the SLIT family proteins that control axonal guidance and branching. Additionally, the tyrosine residues in intracellular carboxyl terminus of SliTrk5 influencing nervous system development and function have a high degree of homology with that of the neurotrophin receptor, tropomyosin-related kinase (Trk) [1, 2]. Scholars identified the SliTrk family proteins originally in a screen for genes that were differentially expressed in the neural tube defects mice [2]. Correspondingly, it has also been verified that six members of the SliTrk family located in three different loci: chromosome 3 (SliTrk3), chromosome 13 (SliTrk1, SliTrk5, and SliTrk6), and the X chromosome (SliTrk2 and SliTrk4) [3], all of which are generally expressed in the developing central nervous system at times and locations that are important to neuronal morphogenesis and synaptogenesis [4, 5], as well as in brain tumors, embryonic stem cells, subsets of endothelial cells, hematopoietic stem cells, and in leukemia and lymphoma cells [6], but vary within the family. For example, SliTrk5 is significantly expressed in the CA1 region of hippocampal [7] and also in occipital and frontal lobes of brain, spinal cord, medulla, and in early hematopoietic progenitors [8, 9], whereas SliTrk1 is expressed in the mature neurons, SliTrk2 is highly expressed in the ventricular layer, and SliTrk6 shows compartmentalized expression in diencephalon. In the vitro experiment, overexpression of SliTrk1 was reported to induce unipolar neurites in cultured neuronal cells but SliTrk5 and other members inhibited neurite outgrowth [10]. Therefore, the members of SliTrk family are not only different in the expression, but also have different functions in the central nervous system. SliTrk5 and its family members regulated the process of synaptogenesis and neurite outgrowth by precisely participating in the formation of synaptic adhesion molecule complexes with the LAR-type receptor phosphotyrosine-phosphatases (LAR-RPTPs) [11–15]. Currently, many investigations have indicated that SliTrk5 may be involved in the pathomechanism of many CNS diseases, including obsessive-compulsive-disorder (OCD), attention deficit/hyperactivity disorder (ADHD), glioma, autism spectrum disorders (ASDs), and Parkinson's disease (PD) [16]. It has also been announced that regulating the expression of SliTrk5 can promote the functional recovery of the nervous system. All these data suggested that SliTrk5 may be involved in the pathogenesis of above diseases and may be an underlying target for the treatment of CNS diseases. Therefore, it is necessary to understand the role of SliTrk5 in the development of the central nervous system and in the pathogenesis of central nervous system diseases.

## 2. Overview of SliTrk5

Exon-mapping using cDNA sequences has revealed the SliTrk5 gene is located in chromosome 13, and there are 8-50 introns in the upstream of initiation methionine, and the protein-coding region of SliTrk5 is located in a single exon. The molecular weight of SliTrk5 predicted by the deduced amino acid sequences is 108.3 kd [7]. SliTrk5 has a characteristic domain architecture consisting of an intracellular carboxy-terminal domain and two consecutive extracellular LRR modules, LRR1 and LRR2. These structures are connected by a single transmembrane domain [6]. The carboxy-terminal regions where conserved tyrosine residues presented are completely conserved between humans and mouse. The homologies of SliTrk5 between mouse and human are 95–97%. Therefore, it can be speculated that the organization and function of the SliTrk5 are similar between human and mouse. All of these results imply that the carboxy-terminal regions and the LRR domain play an important role in the function of SliTrk5 [7]. And it is of great significance to study the molecular structure and function of SliTrk5.

### 2.1. Interaction with Synaptic Adhesion Molecules, RPTP

It has been confirmed that synaptogenesis is an elementary process that establishes definite connections between neurons and supports the organization of neural circuits. In the development of synaptogenesis, the membrane-anchored proteins play a crucial role in initial axon–dendrite target recognition, differentiation of presynaptic and postsynaptic specializations, which called synaptic adhesion molecules (SAMs) [17]. The unique extracellular LRR domain structure of SliTrk5 can combine with the SAMs to control synapse formation, thus regulating the connections between neurons. The LRR domain of SliTrk5 is a typical LRR structure, which contains six LRR repeating motif sandwiched between N-terminal and C-terminal cysteine-rich capping domains, LRRNT and LRRCT, with a defining sequence LxxLxLxxN/GxL (x being any amino acid) [10, 18, 19]. This domain is thought to be homologous to the well-known family of LRR-containing proteins, SLIT family proteins [20], which play a crucial role in axonal guidance and repulsion, tangential neuronal migration, cytoskeletal dynamics, and modifying cell adhesion properties [1, 21]. In addition to SliTrk5, many other leucine-rich neuronal transmembrane proteins have been selected as key synaptic organizers, including LRR transmembrane protein (LRRTM), synaptic adhesion-like molecule (SALM), neurotrophin receptor tyrosine kinase C (TRKC), netrin-G ligand 3 (NGL-3), and fibronectin LRR transmembrane (FLRT) [22–26].

The LRR domain contained in SliTrk5 plays a pivotal role in the regulation of various neuronal functions, such as neurite outgrowth, synapse formation, and dendritic morphogenesis. To execute such functions, SliTrk5 majorly employed the following two basic mechanisms. On the one hand, LRR domain works on the trans cell-cell adhesion molecule PTPRD modulating axon–dendrite adhesion [27, 28], which belong to type IIa receptor protein tyrosine phosphatase (RPTP) family. The RPTP protein family, including PTPRD, PTPRS, and PTPRF, has been shown to be the presynaptic binding partners, interacting with the LRR domain of SliTrks on the postsynaptic membrane to control the formation of inhibitory synapse [29]. In addition, the latest research point of view on structure of synaptic adhesion partner has considered that the binding affinity between RPTP with SliTrks is further modulated by alternative splicing variants (MeA and MeB) in the immunoglobulin-like (Ig-like) domains of RPTP [30, 31]. The crystal structure of the complex formed by the binding of RPTP family proteins with SliTrks reveals the structural basis of its binding mode and the importance of MeB splicing insertion in type IIa RPTP on its binding selectivity and function. Three Ig-like domains of PTPRD bind the LRR1 domain of SliTrks with a 1 : 1 stoichiometry in a MeB splicing insert-dependent manner [11, 32]. Key interaction residues on the type IIa RPTP/SliTrk complex have been shown to be highly conserved in all SliTrk members and type IIa RPTP members, indicating that the binding pattern between PTPRD and SliTrk5 is also similar to the structure described above [12] (Figure 1). Another hand, LRR domain can regulate the function of neuron cell-surface receptor [27, 28]. Song et al. have shown the SliTrk5 acted as a coreceptor of TRKB, regulating brain-derived neurotrophic factor- (BDNF-) dependent biological responses by directly modulating the circulation of TRKB receptor via recruitment of Rab11-FIP3 (an effector protein). They claimed, under normal circumstances, the LRR domain of SliTrk5 interacts primarily with PTPD, whereas it shifts to cis-interactions with TRKB upon the stimulation of BDNF. At this point, PTPD and TRKB compete to combine the LRR domain of SliTrk5 [33]. Therefore, SliTrk5 acts as a common receptor of TRKB, regulating its BDNF-dependent transport and signal transduction in CNS, which plays numerous important roles in synaptic development and plasticity [34]. The LRR domain is the most important structural basis for the function of SliTrk5 in central nervous system.

### 2.2. Function of Tyr Residues in Intracellular Region

Compared with the extracellular LRR domain, the intracellular region of SliTrk5 has a more complex architecture. There are many conserved tyrosine residues in the intracellular region of SliTrk5, which are similar to TRK both in structures and functions, including neurite outgrowth and dendritic elaboration, synapse formation, and neuronal survival [6, 35]. One of the similarities between SiTrk5 and TRK is the presence of NPxY motif (the defining sequence is ASN-Pro-X-TYR, where X is any amino acid) near their intracellular juxtamembrane region [36]. Once phosphorylated, the NPxY motif of TRK could serve as a binding site for adaptor proteins, such as Shc, which initiates Ras and phosphoinositide 3 kinase downstream signal, regulating signal transduction of CNS [37, 38]. In addition, phosphorylation of tyrosine residues in this particular motif has been reported as a signal of receptor endocytosis [39], suggesting that SliTrk5 may recruit Shc or other scaffold proteins to initiate intracellular signal and may be related to endocytosis. Besides, a conserved Tyr residue in a position near the C-terminus that is homologous to that of Y791 structure of TRKA is contained in SliTrk5. The recruitment and activation of the *γ* isoform of phospholipase C (PLC) could be caused by the phosphorylation of Y791 in TRKA, which lead to the decrease of Ca2+ of internal stores and protein kinase C (PKC) activation, finally affecting the transmission of this signal pathway [40–42]. When studying the role of SliTrk5 in vitro HeLa cells, there was another intracellular tyrosine residue (Y833) of SliTrk5 was phosphorylated, which may affect the axon growth [43]. Therefore, we speculate that these conserved tyrosine residues in SliTrk5 may couple to PLC-g signal cascades or other downstream signal proteins, regulating the signal transmission of the CNS.

## 3. Role of SliTrk5 in the Development of CNS

### 3.1. Regulating Neurite Outgrowth and Dendritic Morphology

The function of SliTrk5 in regulating the process of neuronal outgrowth has been established from the beginning. The LRR domain of SliTrk5 is semblable to that of the SLIT family proteins, which are famous for modulating axon guidance and branching [1]. Neurons that overexpressed SliTrk5 have induced more inhibitory input, which potentially decreases neuronal activity and inhibits dendritic growth [44]. In addition, preliminary studies conducted by overexpressing SliTrk5 in PC12 cells showed that compared with the control group, overexpression of SliTrk5 reduced both the number and length of neurites [6]. The Golgi tracing analyses has found in the striatum of adult SliTrk5 deficiency mice; there was a significant decrease in dendritic complexity of medium spiny neurons [16]. In a word, these results suggest that the Slitrk5 is the neuronal components controlling the neurite outgrowth and dendritic morphology.

### 3.2. Promoting Synaptogenesis

There was a study showing that LRR-rich proteins may induce synaptic formation, and the purpose of which was to perform an expression screen for synaptogenesis proteins [45]. SliTrk5 is, as a matter of course, one of those proteins because of its typical LRR domain structure. By immunocytochemical studies in vitro, scholars discovered where the SliTrk5 localized in cultured neurons was on synaptic sites [16]. Moreover, SliTrk5 can not only induce presynaptic neuronal differentiation in cellular coculture system but also promote the formation of inhibitory synapse [44, 46]. Via its extracellular LRR domain, SliTrk5 could bind presynaptic membrane partners, such as PTPRD, and recruit intracellular postsynaptic proteins, participating in the modulation of synapse formation, which has been confirmed [47]. In the process of synapse formation, SliTrk5 was associated with the synaptic adhesion molecules (SAMs), which plays an important role in initial axon–dendrite target recognition, differentiation of presynaptic and postsynaptic specializations. Therefore, SliTrk5 contributes a lot to the development of synaptogenesis, especially the inhibitory synapses.

### 3.3. Affecting the Neuron Survival and Signal Transmission

SliTrk5 has been implicated in promoting neuronal survival. If the SliTrk5 was knocked out, the total brain volume of the mice would be reduced, which was especially obvious in the striatum [16]. Furthermore, researchers have observed the overactivation of the orbitofrontal-subcortical circuits by functional imaging in SliTrk5 knockout mice who exhibited OCD-like behavior, which was posited to be the result of an imbalance of signal transmission in the basal ganglia pathways [48, 49]. In addition, a recent study has demonstrated the ability of SliTrk5 affecting signal transmission in dopaminergic circuits by stimulating the formation of inhibitory synapses in midbrain dopaminergic neurons [44]. In brief, SliTrk5 plays an important role in the survival and signal transmission of neuron.

### 3.4. Participating in Tumorigenesis in Brain

In different types of human brain tumors, the expression of SliTrk5 was most widely in different human brain tumors, compared with other members of the SliTrks family [7]. Especially in the gliomas, the expression of SliTrk5 was upregulated and associated with the pathological grading [50]. In addition to playing an important role in the development of brain tumors, SliTrk5 is also involved in the process of tumorigenesis in other organs, such as colorectal cancer, thyroid tumors, gastric cancer, nasopharyngeal carcinoma, and lung squamous cell carcinoma [51–55]. Thus, besides its role in normal development, SliTrk5 might also be implicated in malignancy.

### 3.5. Involving in Neural Tube Defects

The original cDNA of SliTrk5 and other members of SliTrks were found in a study conducted to identify differentially expressed genes in mice with neural tube defects [6]. Utill now, SliTrk5 is considered to be involved in the mechanism of neural tube defects but the details of their association are still being studied and may be reported elsewhere in the future.

Besides above functions in the CNS, SliTrk5 has also reported to affect the process of angiogenesis and bone formation. A study analysing markers of pork-granulosa cells cultured in vitro found that the expression of SliTrk5 was downregulated over time and proved that SliTrk5 is involved in angiogenesis and vascular development of the ovary, which can be screened as a potential marker [56]. Additionally, SliTrk5 is selectively expressed in osteoblasts and as a negative regulator of hedgehog signal which is necessary for bone formation in osteoblasts. In vitro culture, deletion of SliTrk5 leads to an increase in hedgehog signal, but its overexpression in osteoblasts inhibits downstream targets of hedgehog signal, thus modulating osteoblast differentiation [57]. In a word, SliTrk5 is an emerging protein that is not well understood by people. It plays an important role in diseases of many systems throughout the body, especially in the central nervous system.

## 4. Potential Mechanisms of SliTrk5 in CNS Diseases

SliTrk5 has been identified as one of the factors modulating basic function of the physiological and pathological mechanism of CNS, such as neurite outgrowth, dendritic elaboration, synaptogenesis, and neuronal signal transmission, which was associated to the development of neuropsychiatric disorders, including obsessive-compulsive spectrum disorders (OCDs), attention deficit/hyperactivity disorder (ADHD), autism spectrum disorders (ASDs), and Parkinson's disease (PD) [35].

### 4.1. SliTrk5 in Obsessive-Compulsive Spectrum Disorder (OCD)

Obsessive-compulsive spectrum disorder (OCD), characterized by repeated unwanted thoughts and/or repetitive behavior, is one of the most common mental disorders [58]. Researchers have studied the rare nonsynonymous mutations of the protein-coding sequence of the human SliTrk5 gene in 377 OCD subjects. The results demonstrated that rare functional mutations in SliTrk5 contribute to the impairing of synaptic activity and genetic risk for OCD in human [59, 60]. To study the relationship between SliTrk5 and Tourette's syndrome (TS), which commonly occurs in conjunction with obsessive-compulsive disorder, investigating its role in a family-based sample of 377 affected children, but they did not find any evidence of a link between TS and SliTrk5 [61]. The SliTrk5 deficiency mice whose coding region of the SliTrk5 was replaced by the b-galactosidase gene (lacZ) reporter gene initially showed an increase in anxiety-like behavior (assessed by the elevated-plus-maze and the open-field tests) and followed by repetitive and excessive self-grooming behavior, which eventually lead to severe facial skin damage and hair loss [16]. Excessive grooming that led to the formation of facial lesions, increasing anxiety-like behavior, defects in corticostriatal transmission, and altered expression of glutamate receptors in the striatum, and all of these behavior and pathway manifestation found in the SliTrk5 deficiency mice are similar to another genetic mouse model of OCD which has been reported lacking the synapse-associated protein 90-postsynaptic density-95-associated protein 3 (Sapap3) [62]. Sapap3 is an intracellular scaffolding molecule localized to the postsynaptic position of excitatory synapses and is crucial for maintenance of synaptic structure [63, 64]. In addition, another mouse model of OCD with repetitive grooming behavior was Hoxb8 deficiency mice, which was almost identical to that observed in SliTrk5 deficiency mice [65–67]. However, the treatment of fluoxetine, as a selective serotonin reuptake inhibitor (SSRI), which is mainly used for the treatment of depression and obsessive-compulsive disorder, can effectively alleviate reduce the excessive grooming behavior of SliTrk5 deficiency mice [68]. Because the SliTrk5 intracellular domain resembles TRK neurotrophin receptors, it is plausible that they may have similar ligands. It would be interesting because neurotrophin can be modulated by existing drugs such as FLX [69]. Meanwhile, FLX can alleviate the obsessive-compulsive like behavior in SliTrk5-deficient mice. All of above evidences suggested that the expression or the activity of SliTrk5 may be regulated by FLX, but it is still obscure. Future studies that investigate the disease relevance of the human gene are essential for SliTrk5 to emerge as an important therapeutic target and/or biomarker for OCD [70].

The possible pathological mechanisms of SliTrk5 in OCD include the following:

1. Affecting the anatomy of striatum

The effect of SliTrk5 on the anatomy of striatum mainly contains two aspects. Firstly, the volume of the striatum was reduced in both young and aged mice whose SliTrk5 gene has been knocked out. The striatum volume relative to the whole brain estimated by Cavalieri measuring showed a significant decrease in striatum volume compared with wild-type mice, while the ratio of other brain structures to total brain volume did not change, suggesting that SliTrk5 deficiency significantly affected the anatomical structure of the striatum [16]. These results found in SliTrk5 deficiency mice, in line with many previous studies, reported that the volume of the striatum is decreased, as well as in some but not all individuals with OCD [71–73]. Secondly, it has been revealed that there was a significant decrease in dendritic complexity at 50 *μ*m and greater distance from the soma in the individual medium spiny neurons of the striatum in Slitrk5 deficiency mice, either using the Sholl analysis to observe the dendritic complexity or using fractal dimension analysis to quantify how completely a neuron fills its dendritic field, all of which has reflected a decrease in synaptic connectivity. However, there was no difference in striatal cell soma area between SliTrk5 deficiency mice and their wild-type litter born larva [16]. In conclusion, it is possible the lessened striatal volume in the SliTrk5 deficiency mice might be accounted for by altered neuronal morphology (Table 1).

(2) Increasing the orbitofrontal cortex activity

To investigate the role of SliTrk5 in the central nervous system, scholars evaluated the difference of baseline activity in specific brain regions between wild-type and SliTrk5 knockout mice by assessing expression of FosB, which is a transcription factor used to assess neuronal activity routinely. As a result, they found that FosB was upregulated exclusively in the orbitofrontal cortex of SliTrk5 knockout mice, which did not show in other brain regions [16, 74]. This finding also has been consistently verified in functional imaging studies that discovered there is an increasing activity in orbitofrontal cortex in individuals with OCD (Table 1) [49, 75].

(3) Modulating region-specific glutamatergic neurotransmission

Shmelkov et al. have discovered the protein amounts of glutamate receptor subunits NAMDAR2A, NAMDAR2B, Glutamate Receptor-1, and Glutamate Receptor-2 involved in excitatory neurotransmission were decreased by 20–60% in SliTrk5 deficiency mice, greatly modulating the glutamatergic neurotransmission of specific region [16].The sequence variation of SliTrk5 was also considered may be associated with the structural neuroimaging phenotype of obsessive-compulsive disorder [76]. Probably because of these defects, the corticostriatal neurotransmission of SliTrk5 deficiency mice was impaired, agreeing with the observation of altered corticostriatal transmission in OCD patients [77, 78]. Current studies have highlighted the important role of excitatory synapses in the striatum and cortical striatum nerve conduction in the pathogenesis of OCD-like behavior (Table 1) [79]. Consequently, SliTrk5 may be involved in the pathogenesis of OCD by regulating the glutamatergic neurotransmission, thus affecting the corticostriatal neurotransmission.

### 4.2. SliTrk5 in Brain Tumor

Recent years, SliTrk5 was reported to participate in the development of brain tumors. A previous study has validated the expression of SliTrk5 is most widely expressed in different brain tumors, which was upregulated in gliomas and correlated with pathological grading [7, 50]. SliTrk5 can promote BDNF-dependent signal by acting as a TRKB coreceptor in striatum neurons [33]. Brain-derived neurotrophic factor (BDNF) is widely distributed in the central nervous system, affecting the malignant degree of glioma [80]. BDNF can inhibit neuronal apoptosis through its functional receptor TRKB. In neurocytoma, BDNF can induce TRKB phosphorylation, activating Ras/ERK signal transduction pathway and promoting cell proliferation [81, 82]. Some studies have shown that the activation of TRKB-BDNF signal pathway can promote nerve cells to synthesize and secrete vascular endothelial growth factor(VEGF), thus promoting the growth of tumor cells [83, 84].Therefore, some researchers have speculated that SliTrk5 may stimulate the occurrence and proliferation of glioma by modulating TRKB-BDNF signal pathway and other related signal transduction.

SliTrk5 is also associated with tumorigenesis in other organs. SliTrk5 gene presented frequent genetic, epigenetic, and transcriptional alterations in colorectal neoplasia, which has been discovered by a study designed to compare and contrast the molecular profiles of laterally spreading tumors (LSTs) and colorectal cancer (CRC) [51]. Moreover, in thyroid tissue, the expression of SliTrk5 was significantly downregulated in Trk-T1 transgenic thyroid tumor mice, which was revealed by a global genomic copy number analysis [52]. SliTrk5 also has been identified affecting the molecular or clinical phenotypes of gastric cancer (GC) with TP53 mutation [53] and correlating with the radioresistance of nasopharyngeal carcinoma and the prognosis of lung squamous cell carcinoma (Table 1) [54, 55].

SliTrk5 is not only involved in the tumorigenesis of the central nervous system but also related to tumors of all systems of the whole body, in which there may be some underlying common mechanisms. If we take SliTrk5 as a target for antitumor therapy in the future, there may be some unexpected surprises.

### 4.3. SliTrk5 in Attention Deficit/Hyperactivity Disorder (ADHD)

The main symptoms of ADHD are inattention and/or hyperactivity/impulsivity, and SliTrk5 can regulate the hyperactivity behavior of ADHD by controlling the formation of inhibitory synapses in dopamine neurons [44]. The possible mechanisms are as follows: the neurodevelopmental of the hyperactivity disorder has been discovered to be involved in the dopaminergic neurons system, and SliTrk5 was identified to promote inhibitory synapse formation on midbrain dopaminergic neurons, whereas SliTrk2 has opposite effects. Loss of the function of SliTrk2 results in less excitatory input and hyperactivity, but loss of SliTrk5 function results in less inhibitory input and locomotor activity. Both of them would cause the imbalance of excitatory/inhibitory synaptic, leading to alterations in developing dopaminergic circuits and significantly affecting locomotor activity, which has also been identified to disrupt neurotransmission of dopaminergic neurons and contribute to many neuropsychiatric disorders including hyperactivity disorder (Table 1) [44, 85]. If we can control the balance of excitatory and inhibitory synapses by targeting the relative expression levels of SliTrk5 and SliTrk2, the symptoms of ADHD may be improved to some extent.

### 4.4. SliTrk5 in Autism-Spectrum-Disorders (ASDs)

The autism spectrum disorder (ASD) is characterized as restricted repetitive behavior, including the lower-order stereotypy and self-injury and higher-order indices of circumscribed interests and cognitive rigidity [86]. A genome comparison study designed to identify related genes for autism has found that the SliTrk5 is associated with repeated overgrooming of ASDs (Table 1) [87]. Thus, although no study has identified a specific role of SliTrk5 in the pathogenic mechanism of autism so far, SliTrk5 may be one of the genetic factors of autism from a genetic point of view. Targeting studies of SliTrk5 are needed in autism in the future.

### 4.5. SliTrk5 in Parkinson's Disease (PD)

SliTrk5 can effectively reclaim activated TRKB receptors and promote BDNF-dependent signal pathway, prolonging the intensity and duration of neurotrophic factor signal in striatum neurons in the absence of BDNF supply [33]. Moreover, the SliTrk5 deficiency mice showed that striatum volume and anatomical structure were changed [16]. The striatum is the largest component of the basal ganglia, and the disorder of striatal function has been implicated in neurodegenerative disorders such as Huntington's disease and Parkinson's disease [88, 89]. Additionally, SliTrk5 can be regulated by Lmx1(a/b), which as a transcription factor involved in each step of midbrain dopaminergic neuron development [90, 91]. The specific inactivation of Lmx1(a/b) in adult midbrain dopaminergic neuron resulted in dopamine neuron degeneration and parkinsonism [91, 92]. Although no current researches have shown that there is a clear relationship between SliTrk5 and these neurodegenerative diseases, SliTrk5 may affect the function of midbrain dopaminergic neurons through above pathways, leading to neurodegenerative diseases such as Parkinson's disease. And SliTrk5 has represented a new potential target of therapeutics for these neurodegenerative disorders by enhancing interaction with TRKB receptors in the absence of exogenous neurotrophic factors or regulating the function of striatal neurons (Table 1).

## 5. Summary

Increasing evidence has revealed that SliTrk5 plays an important role in the physiological and pathological processes of the CNS. The neurite outgrowth, dendritic branching, synaptogenesis, cell differentiation, and signal transmission of neurons are important processes for the development of CNS. SliTrk5 is an important synaptic associated protein that has a crucial regulatory effect on the above response processes of CNS. Furthermore, there have been exhibiting complex interactions between SliTrk5 and many CNS disorders, including obsessive-compulsive disorder, attention deficit/hyperactivity disorder, autism spectrum disorders, and brain gliomas. The role of SliTrk5 in the neurodegenerative diseases, such as Parkinson's disease, has been starting to come out. Taking SliTrk5 as the target and regulating its expression can alleviate neural function damage and promote the recovery of neural function, suggesting that SliTrk5 may be a promising target molecule for illustrating the mechanisms and the treatment of CNS diseases (Table 1). As the specific pathogenesis and signal pathway of SliTrk5 in CNS diseases are not fully clear, the randomized controlled clinical trials need to take years to conduct. Thus, this review has provided the foundation for subsequent integrated studies into the treatment of CNS disorders by figuring out the various functional roles of SliTrk5 in terms of the development of CNS. The specific relationship and potential mechanism between SliTrk5 and neurodegenerative diseases will also be the focus and trend of future research. Consequently, SliTrk5 very likely plays a crucial role in the development of CNS diseases by regulating synaptogenesis and other physiological mechanisms.

## Figures and Tables

**Figure 1:** Functional structure of SliTrks and cell adhesion molecule IIa receptor protein tyrosine phosphatases (RPTPs) and their interaction in synapse formation.

**Table 1:** Possible mechanisms of SliTrk5 in CNS diseases. OCD: obsessive-compulsive-disorder; ADHD: attention deficit/hyperactivity disorder; ASDs: autism spectrum disorders; PD: Parkinson's disease.

Disease	Expression site of SliTrk5	Possible mechanisms	Participants or models	Potential therapeutic target
OCD	Cortical striatum	(1) Affecting the anatomy of striatum (2) Increasing the orbitofrontal cortex activity (3) Modulating region-specific glutamatergic neurotransmission	SliTrk5 knockout mice	SSRI fluoxetine (FLX) can alleviate the OCD-like behaviors in mice, including excessive self-grooming and anxiety-like behaviors.
Brain tumor	Upregulating expression in gliomas	SliTrk5 may stimulate the occurrence and development of glioma by mediating TRKB-BDNF signal pathway and other related signal transduction.	Patients with glioma	SliTrk5 gene targeting therapy may be the trend in the future.
ADHD	Midbrain dopaminergic neurons	SliTrk5 can modulate the hyperactivity behavior of ADHD through promoting inhibitory synapses formation on midbrain dopaminergic neurons.	SliTrk5 knockdown mice	Regulating the expression of SliTrk5 can maintain the balance of excitatory/inhibitory synapse signal transmission.
ASDs	Unknown	Genetic factors	ASD mice models	SliTrk5 gene targeting therapy may be the trend in the future.
PD	Unknown	Affecting the function of midbrain dopaminergic neuron	/	Enhancing interaction of TRKB receptors with SliTrk5 in the absence of exogenous neurotrophic factors or regulating the function of striatal neurons maybe a new potential target for therapeutics of PD.
